# L-Plastin Nanobodies Perturb Matrix Degradation, Podosome Formation, Stability and Lifetime in THP-1 Macrophages

This article has been retracted.

**DOI:** 10.1371/journal.pone.0078108

**Published:** 2013-11-13

**Authors:** Sarah De Clercq, Ciska Boucherie, Joël Vandekerckhove, Jan Gettemans, Aude Guillabert

**Affiliations:** Department of Biochemistry, Ghent University, Faculty of Medicine and Health Sciences, Ghent, Belgium; West Virginia University, United States of America

## Abstract

Podosomes are cellular structures acting as degradation ‘hot-spots’ in monocytic cells. They appear as dot-like structures at the ventral cell surface, enriched in F-actin and actin regulators, including gelsolin and L-plastin. Gelsolin is an ubiquitous severing and capping protein, whereas L-plastin is a leukocyte-specific actin bundling protein. The presence of the capping protein CapG in podosomes has not yet been investigated. We used an innovative approach to investigate the role of these proteins in macrophage podosomes by means of nanobodies or Camelid single domain antibodies. Nanobodies directed against distinct domains of gelsolin, L-plastin or CapG were stably expressed in macrophage-like THP-1 cells. CapG was not enriched in podosomes. Gelsolin nanobodies had no effect on podosome formation or function but proved very effective in tracing distinct gelsolin populations. One gelsolin nanobody specifically targets actin-bound gelsolin and was effectively enriched in podosomes. A gelsolin nanobody that blocks gelsolin-G-actin interaction was not enriched in podosomes demonstrating that the calcium-activated and actin-bound conformation of gelsolin is a constituent of podosomes. THP-1 cells expressing inhibitory L-plastin nanobodies were hampered in their ability to form stable podosomes. Nanobodies did not perturb Ser5 phosphorylation of L-plastin although phosphorylated L-plastin was highly enriched in podosomes. Furthermore, nanobody-induced inhibition of L-plastin function gave rise to an irregular and unstable actin turnover of podosomes, resulting in diminished degradation of the underlying matrix. Altogether these results indicate that L-plastin is indispensable for podosome formation and function in macrophages.

## Introduction

Podosomes are cellular structures which establish close contact with the extracellular matrix. They were discovered in monocytic cells such as macrophages, dendritic cells and osteoclasts [1]–[3]. More recently, other cell types such as endothelial cells and smooth muscle cells have been shown to form podosomes upon stimulation with cytokines [4], [5] or phorbol esters [6], [7]. Similar structures are found in cancer cells, termed ‘invadopodia’ [8].

Usually situated at the periphery of the cellular membrane, podosomes display a polarized distribution pattern in migrating cells, located between the lamellipodium and lamellum [9]. Their primary purpose is connected to cellular motility, matrix remodeling and tissue invasion. Therefore, they are highly dynamic structures and are mainly found in motile cells that have to cross tissue boundaries [10]. Podosomes are physiologically relevant structures, as impairment of podosome formation leads to a number of symptoms and diseases. A most notable example is the Wiskott-Aldrich syndrome (WAS), arising due to mutations in the gene encoding WASP (important in podosome formation), and characterized by immune defects, eczema and lymphoma [11].

Podosomes present as dot-like structures (0.5–2 µm diameter) at the ventral cell surface, and consist of a central ‘core’ rich in tightly packed actin bundles, surrounded by a ring of adhesion, signaling and scaffolding proteins including, among others, integrins, talin, paxillin and vinculin. The actin core is connected to the ring domain by an array of radial actin fibers, which ancor the core bundle to the ring [12]. The core bundle of podosomes is enriched in several actin-associated proteins, such as Arp2/3, cortactin, WIP, WASP, dynamin and gelsolin [10]. The filaments within these structures are highly regulated by actin nucleators, crosslinking proteins, kinases and small GTPases. Consequently, total actin turnover occurs within seconds [2].

This study focuses on 3 well-known actin binding proteins: L-plastin, gelsolin and CapG. L-plastin or “leukocyte-plastin” (LPL) occurs predominantly in hematopoietic cells, but ectopic expression is also observed in cancer cells [13], [14]. Bundling proteins like L-plastin bind 2 actin filaments and cross-link them into tight bundles. LPL is composed of 2 N-terminal EF-hands, involved in calcium binding, followed by 2 actin binding domains (ABDs). Its F-actin binding and bundling activities are negatively regulated by calcium [15]. L-plastin contains two N-terminal phosphorylation sites: Ser5 (predominant site) and Ser7. Phosphorylation enhances targeting of LPL to F-actin rich structures and increases its actin bundling activity [16]. Gelsolin and CapG are members of the gelsolin superfamily. Gelsolin consists of 6 homologous structural domains, whereas CapG has only 3 such domains [17]. They are both widely expressed in mammalian cells, including hematopoietic cells such as neutrophils and macrophages [18]–[21]. Gelsolin severs F-actin after which it remains attached to the barbed end of the filament as a cap, preventing further actin polymerization. CapG shares this capping function with gelsolin, but lacks its severing function [22], [23]. They are both activated by calcium and negatively regulated by phosphoinositides, and both are involved in organizing cell structure, motility and invasion [21], [24]–[28].

L-plastin and gelsolin (GSN) have both been shown to reside in podosomes. L-plastin function in podosomes has not been fully elucidated yet, but it probably plays a role during early stages of cell adhesion and spreading. The presence of gelsolin in podosomes has been well documented [29]–[31]. In GSN−/− osteoclasts the formation and degradative activity of podosomes is impaired [30], whereas in dendritic cells, gelsolin deficiency does not affect podosome formation and function [32]. The presence of CapG in podosomes has not been investigated yet.

Nanobodies correspond with the antigen-binding domains of “heavy-chain only antibodies”, which are found in *Camelidae* species and cartilaginous fish such as sharks [33], [34]. They are only 15 kDa in size and can be easily cloned. Nanobodies generally bind their target with nanomolar affinity and have been used in a number of applications: neutralization of toxins [35], as a crystallization aid [36], inactivation of viral proteins [37], or blocking selected functions of cytoskeletal proteins in the cytoplasm [38]–[40].

In this study we used *bona fide* nanobodies against L-plastin, gelsolin and CapG as intrabodies to investigate if, and to what extent, these functionally distinct proteins contribute to podosome function and integrity. The majority of nanobodies that were used inhibit biochemical activities of their target, resulting in a protein domain ‘knock-out’, without affecting their expression level in cells. We report that expression of L-plastin nanobodies in macrophage-like THP-1 cells perturbs podosome formation and stability, as evidenced by a higher turn-over, and concurrent shorter lifetime, of podosomes. In addition, blocking L-plastin bundling or locking L-plastin in an inactive conformation reduces the ability of these cells to degrade the extracellular matrix. We further demonstrate that phosphorylated L-plastin is highly enriched in podosomes, underscoring the importance of its actin bundling properties in podosome stability. Gelsolin and CapG nanobodies on the other hand, did not significantly affect podosome formation or matrix degradation. Hence, L-plastin is an integral and functional constituent of macrophage podosomes.

## Results

### Unlike CapG, L-plastin and gelsolin localize in podosomes of macrophage-differentiated THP-1 cells

The composition and assembly of podosomes have been under extensive research (reviewed in [10], [31], [41]). Several actin binding proteins are present in podosomes, but for some, their exact functions have not been elucidated. Nanobodies targeting functional regions of such proteins with nanomolar affinity serve as a tool to investigate protein function(s) in distinct cellular contexts, as demonstrated before [38]–[40] (Van Impe et al, unpublished data). The presence of CapG in podosomes has not been investigated yet, but L-plastin and gelsolin were shown to reside in podosomes (reviewed in [10], [31], [41], [42]). We set out to employ nanobodies against these constituents in the podosome assembly process in macrophage-like THP-1 cells.

THP-1 cells, a human monocytic leukemia cell line, are one of the most widely used models to study the monocytic differentiation process and biological functions of differentiated cells [43], [44]. They grow in suspension but can be easily differentiated into adherent macrophage-like cells by treatment with compounds such as phorbol-12-myristate-13-acetate (PMA) [45], [46]. Following treatment with PMA, these cells constitutively form podosomes [47], [48]. Indeed, stimulation with PMA for 3 days promoted formation of actin-rich podosomes in most of the cells and both L-plastin and gelsolin were enriched in these podosomes, in contrast to CapG (Fig. 1A). We determined the intensity profiles of F-actin and L-plastin, gelsolin or CapG along a line intersecting the whole cell. The podosome is defined as an area that is highly enriched in F-actin, defined here as an increased F-actin staining intensity. The intensity profiles emphasize that gelsolin and L-plastin coalesce with F-actin enriched structures, meaning they are enriched in podosomes, while CapG shows a more diffuse and distinct staining pattern (Fig. 1B).

**Figure 1:** L-plastin and gelsolin localize to podosomes of THP-1 macrophages. (A) Monocytic THP-1 cells were differentiated with PMA for 3 days. Cells were stained for F-actin (phalloidin-alexa 594, red) and L-plastin, gelsolin or CapG (alexa-488, green). The pictures were acquired with a laser scanning confocal microscope and are representative for three independent experiments. Bar: 10 µm. (B) Graph of the F-actin and LPL/CapG/GSN intensities measured along the line, drawn across the (podosomes of the) cell. Intensity profiles were represented as function of the length (µm) of the line. (C) Lysates of PMA-stimulated versus –unstimulated THP-1 cells were blotted and probed for L-plastin, CapG, actin or gelsolin. Blots are representative for two independent experiments. Densitometry was used to determine band intensity in (C) and is expressed as GSN:actin, LPL:actin and CapG:actin.

Interestingly, the L-plastin and gelsolin expression level increases as judged by western blotting on crude lysates of PMA-stimulated THP-1 cells (Fig. 1C). The expression was 2.5–3 fold higher after PMA stimulation, whereas there was no difference in CapG expression between stimulated and unstimulated cells. Our data indicate that L-plastin and gelsolin are *bona fide* constituents of podosomes in THP-1 cells.

### Actin-bound gelsolin is enriched in podosomes whereas LPL Nbs target actin-free L-plastin

We expressed EGFP-tagged L-plastin, gelsolin or CapG nanobodies (Fig. 2A) in macrophage-like THP-1 cells in a stable manner by lentiviral transduction. L-plastin nanobody 5 (LPL Nb5) blocks the actin bundling activity by targeting a hinge region in between the actin binding domains of L-plastin (K_d_ 40 nM). L-plastin nanobody 9 (LPL Nb9) interacts with the N-terminal EF-hands (K_d_ 80 nM) in a calcium-dependent manner and locks plastin in an inactive conformation [39] (Fig. 2A). Gelsolin nanobody 11 (GSN Nb11) prevents gelsolin-G-actin interaction (K_d_ 5 nM) irrespective of the calcium concentration whereas GSN Nb13 only recognizes calcium-activated gelsolin (K_d_ 10 nM) [40]. CapG Nb4 binds to the first domain of CapG (K_d_ 5.3 nM), but has no inhibitory effect on F-actin or G-actin binding by CapG (Van Impe et al., unpublished data). Immunoprecipitation experiments confirmed the efficacy of nanobodies to pull-down their respective antigens, following expression induction with doxycycline (0.5 µg/ml) (Fig. 2B). Expression of LPL Nb5 and GSN Nb11 was higher as compared to LPL Nb9 and GSN Nb13, respectively, as observed previously in Jurkat T cells [38]. In THP-1 cells, the LPL nanobodies interacted with L-plastin that was completely devoid of actin as observed previously [39] whereas GSN nanobodies bound two different gelsolin populations, in agreement with earlier observations [40] (Fig. 2C). These findings highlight consistent nanobody functionality in different cell types. Actin did not co-immunoprecipitate with CapG Nb4 (Fig. 2C).

**Figure 2:** Nbs targeting distinct structural domains of L-plastin, gelsolin and CapG, interact specifically with their target. (A) LPL consists of two N-terminally located EF-hands (EF) and two C-terminally located ABDs. Both ABDs are divided into two calponin homology (CH) domains. LPL Nb9 recognizes the EF-hands, whereas LPL Nb5 binds the two ABDs combined. Gelsolin consists of six homologous domains, whereas CapG consists of 3 domains. GSN Nb11 recognizes the N-terminal part (domain 2) and GSN Nb13 binds to domains 4 and 5 combined (C-terminal part). CapG Nb4 binds to the first domain of its target. (B) THP-1 cells expressing EGFP-tagged LPL/GSN/CapG Nbs or EGFP were generated by stable transduction; expression of these constructs is induced by doxycycline. Cell lysates were incubated with a polyclonal EGFP antibody, followed by binding on protein G sepharose to immunoprecipitate the EGFP-tagged Nbs or EGFP. The blots were stained for L-plastin, gelsolin or CapG and EGFP to demonstrate the interaction between the expressed Nb and its target in the presence of doxycycline. (C) Co-immunoprecipitations experiments as described in (B) were conducted in the absence or presence of EGTA. The blots were stained for L-plastin, gelsolin or CapG, EGFP and actin. Blots are representative for four independent experiments. CL: crude lysate, DOX: doxycycline.

Considering their localization and biological properties, GSN and L-plastin likely participate in dynamic actin reorganization during podosome formation and/or disintegration but mechanistic insights are lacking. To check whether GSN and LPL nanobodies are targeted to podosomes and interact with their respective antigens, we investigated their subcellular localization in THP-1 cells. Cells stably expressing EGFP or EGFP-tagged CapG Nb4 were used as negative controls and were therefore also stained for L-plastin. Notably, GSN Nb13 was enriched in podosomes (Fig. 3) and the intensity profile confirmed that GSN Nb13 coincided with the profile of actin and gelsolin (Fig. S1). For GSN Nb11, this was not the case. These results are in agreement with immunoprecipitation experiments (Fig. 2C) [38], [40]. LPL Nb5 and 9 were mostly not enriched in podosomes (Fig. 3) and this is in accordance with previous data showing that LPL Nbs recognize an actin-free population of LPL (Nb9) or prevent actin bundling (Nb5) [38]. This is underscored by immunoprecipitation experiments (Fig. 2C). The observed intensity profile is diffuse, contrasting with F-actin but similar to the pattern of EGFP and CapG Nb4 (Fig. S1). We conclude that GSN Nb13 targets calcium-activated and actin-bound gelsolin and traces this complex in podosomes, indicating that endogenous gelsolin is a *bona fide* component of podosomes in THP-1 cells. We next investigated potential defects in podosome function induced by nanobodies.

**Figure 3:** L-plastin Nbs perturb podosome formation in PMA-stimulated THP-1 cells. Cells were incubated with PMA for 72-tagged LPL/CapG/GSN Nbs or EGFP was induced by 24 hr incubation with doxycycline (0.5 µg/ml). Cells were stained for F-actin (phalloidin 670, far red, shown in grey) and L-plastin or gelsolin (alexa-594, red). EGFP and EGFP-tagged nanobodies are shown in green. The pictures were acquired with a confocal laser scanning microscope and are representative for four independent experiments. Bar: 10 µm.

### Gelatin degradation by THP-1 cells is impaired by LPL nanobodies

Podosomes are thought to contribute to tissue invasion and matrix remodeling. Invadopodia have been recognized early on as structures that degrade matrix proteins [49] whereas for podosomes this was demonstrated more recently [50]. We plated cells onto Cy3-labeled gelatin-coated coverslips for 24 hours. Matrix degradation was observed as black areas (Fig. 4A). 30%–35% of THP-1 cells expressing EGFP, CapG Nb4, GSN Nb11 or 13 degraded the matrix within 24 hours (Fig. 4B). For cells expressing LPL Nb5, only 18.7% of the cells degraded the matrix. For LPL Nb9-expressing cells, this number was further reduced to 11.9%. Thus L-plastin is specifically involved in matrix remodeling and LPL Nbs counteract the function of L-plastin in podosomes of THP-1 cells whereas GSN and CapG Nbs have no such effect.

**Figure 4:** LPL Nbs impair gelatin degradation by THP-1 cells but MMP production and secretion remain unaffected. THP-1 cells were plated onto Cy3-labeled gelatin-coated glass coverslips for 24 hours and subjected to immunofluorescence analysis. (A) EGFP-tagged nanobodies are depicted in green and gelatin in red. In the merged pictures, the nuclei are stained by DAPI and depicted in blue. Dark regions in the fluorescent gelatin monolayer (red) are indicative of gelatin degradation. Bar: 30 µm. (B) Quantification of the percentage of THP-1 cells capable of degrading the gelatin matrix. Data indicate means +/− SEM from 3 independent experiments (n = 450–800). Unpaired t-tests were performed to observe statistical differences in the degradation potential between cells expressing EGFP and cells expressing the nanobodies (ns: non significant p>0.05; ** p<0.01; *** p<0.001). Stably transduced THP-1 cells (5×10^5^ cells per condition) were seeded into 12-wells in the presence of PMA for 72 h. (C) The conditioned media of these cells were subjected to gelatin zymography. (D, E) Immunoblot analysis performed on THP-1 cell lysates (D) and conditioned media (E) for (pro-)MMP2, (pro-)MMP9,(pro-)MMP14 (D) and (pro-)MMP9 respectively (E). In (D), actin was used as a loading control. These data are representative of 8 independent experiments.

### The decrease in matrix degradation efficiency for LPL Nbs is independent of MMP production, secretion or localization

Degradation of the extracellulair matrix by podosomes occurs by localized secretion of specialized proteases [51]. We set out to examine whether the low matrix degrading capacity of LPL Nb-expressing THP-1 cells could result from altered expression, release and/or localization of matrix-degrading proteases. Matrix metalloproteinases (MMPs) are known to be important for matrix degradation by podosomes and invadopodia (reviewed in [51], [52]). MMP2, MMP9 and MMP14 belong to the ‘standard equipment’ of podosomes and invadopodia [41], [51] and are by consequence the most studied representatives in macrophages and other podosome-displaying cells. These MMPs are secreted in an inactive (latent) form, called zymogen or pro-MMP. Latent MMPs require activation to become active enzymes able to cleave ECM components. MMP2 and MMP9 are gelatinases, whereas MMP14 is a membrane-type matrix metalloproteinase (MT1-MMP). Especially MMP9 (pro-MMP9) is extensively expressed in and secreted by macrophages [53].

To test a possible role for L-plastin in the secretion of MMPs, we performed gelatin zymography on conditioned media of stable THP-1 cells. The results in Fig. 4C show that MMP9, based on its gelatinase activity and apparent molecular weight, indeed is the most prominent protease in (THP-1) macrophages. When cells were seeded on fibronectin-coated wells, the secretion of (pro-)MMP2 (pro-MMP2: 72 kDa/MMP2: 64 kDa) increased slightly (Fig. S2A), which has also been reported for dendritic cells [54] and T lymphocytes [55]. However, secretion of (pro-)MMP9 and (pro-)MMP2 in LPL Nb-expressing THP-1 cells was not reduced compared to control conditions or other nanobodies (Fig. 4C and Fig. S2A). Immunoblot analysis of the corresponding cell lysates (Fig. 4D: MMP2 and MMP9) and media (Fig. 4E: MMP9 and Fig. S2B: MMP2) showed that production of these MMPs was the same for all conditions, which is in agreement with the results shown in Fig. 4C. Again, MMP2 could only be detected in conditioned medium when the cells had been stimulated with fibronectin (Fig. S2B). MMP14 or MT1-MMP was also detected in cell lysates but expression of this protease was similar for the different nanobodies and EGFP (Fig. 4D).

Microscopic analysis of the localization of MMP2, MMP9 and MMP14 in parental THP-1 cells confirmed that MMP9 is a highly expressed protease (Fig. S2C). Stable macrophage-like THP-1 cells were also stained for MMP2, MMP9 and MMP14. The localization and expression of MMP9 (Fig. S2D), MMP2 and MMP14 (data not shown) did not change in LPL-Nb expressing THP-1 cells. Taken together, these results indicate that the low degrading capacity of LPL Nb-expressing THP-1 cells is not due to altered proteolytic activity. We also conclude that only LPL Nbs perturb functional podosome formation while others seem to have little or no affect at all. We therefore further examined the underlying mechanism.

### Ser5 phosphorylated L-plastin localizes to podosomes

L-plastin phosphorylation increases its F-actin bundling activity and promotes targeting to sites of actin assembly in the cell by switching the protein from a ‘low-activity’ to ‘high-activity’ state [16]. We previously demonstrated the importance of LPL Ser5 phosphorylation upon CD3/CD28-activation of human T-cells [38]. We first investigated the localization of phosphorylated L-plastin in PMA-stimulated macrophage-like THP-1 cells using a Ser5 phospho-L-plastin antibody [16]. A striking focal enrichment of phosphorylated L-plastin in podosomes could be observed in these cells (Fig. 5A). Secondly, we investigated whether phosphorylation of LPL in PMA-stimulated THP-1 cells that express LPL Nb5 or 9 is affected. Interestingly, whereas L-plastin nanobodies delay and reduce L-plastin phosphorylation in CD3/CD28-stimulated Jurkat T cells [38], the level of phosphorylation and kinetics were unaffected in THP-1 cells (Fig. 5B). A drastic increase in LPL phosphorylation was observed after 15 min with a maximum at 30–45 min. After one hour of PMA treatment the signal decreased. This pattern is conserved for the different stable THP-1 cells indicating that the observed effects on matrix remodeling is independent of the L-plastin phosphorylation status and that L-plastin phosphorylation is dependent on the cell context.

**Figure 5:** Ser5 phosporylated L-plastin is enriched in podosomes. (A) PMA differentiated THP-1 cells were stained for phospho-Ser5 L-plastin (alexa 488, green) and F-actin (phalloidin-alexa 594, red). Bar: 10 µm. (B) L-plastin phosphorylation is unaffected by LPL Nbs. THP-1 cells stably expressing EGFP, GSN Nb11, LPL Nb5 and LPL Nb9 were stimulated for different periods of time with PMA. The blots were stained for phospho-L-plastin and total L-plastin as a loading control. Data are representative of three independent experiments. Densitometry was used to determine band intensity in (B) and is expressed as phospho-LPL:LPL.

### L-plastin nanobodies perturb podosome formation in THP-1 cells

Close examination of THP-1 cells expressing LPL Nb5 or 9 revealed striking effects since the distinct, ‘dot-like’ appearance of actin and cortactin, which is so typical for podosomes, disappeared in many of the observed cells. This is shown for LPL Nb5 in Fig. 6A (actin staining) and Fig. S3 (actin/cortactin staining). This finding was unique to L-plastin nanobodies and could not be observed for THP-1 cells expressing EGFP, CapG Nb4 or GSN nanobodies, again attesting to the specificity. For LPL Nb5/9, podosomes did not present as crisp, distinct dots, but many cells showed a diffuse phenotype with blurry dots. We term this a ‘disrupted phenotype’ and quantified as such the number of cells that showed ‘normal podosomes’, ‘no podosomes’ or the ‘disrupted phenotype’ (Fig. 6B). LPL Nb5- and Nb9-expressing cells showed significantly more cells with a disrupted phenotype (43.57% and 40.04%, respectively, compared to ±20% for EGFP-, CapG Nb4- and GSN Nb-expressing cells). The number of cells displaying normal podosomes was significantly decreased for cells expressing LPL Nb5 (23.42%) or LPL Nb9 (31.92%) compared to other conditions (50–60%). There was also a significant increase in cells that lack podosomes for LPL Nb5 (33.02%) compared to other conditions (18–28%). Moreover, staining of LPL in the LPL Nb-expressing cells revealed also a diffuse, ‘disrupted’ phenotype, coinciding with the F-actin pattern (Fig. 3), or LPL being even completely absent from podosomes (Fig. 6C). We therefore reasoned that LPL Nbs may trigger podosome instability by disrupting L-plastin F-actin bundling activity (Nb5) or preventing its activation (Nb9). To verify this hypothesis we visualized and quantified the lifetime of podosomes.

**Figure 6:** LPL Nbs disturb podosome integrity. (A) Confocal images showing the different phenotypes, observed in THP-1 macrophages. Cells expressing GSN Nb11 or LPL Nb5 are shown in green and cells were stained for F-actin (phalloidin-alexa 594, red). Bar: 10 µm. (B) Representation of the observed phenotypes (‘Podosomes’, ‘No podosomes’ and ‘Disrupted phenotype’) for the different constructs. 600–1200 cells were counted per condition in 4–5 independent experiments. Error bars represent mean ± SEM. Unpaired t-tests were performed to observe statistical differences between cells expressing EGFP and cells expressing the nanobodies (ns: non significant p>0.05; * p<0.05). (C) THP-1 macrophages stably expressing LPL nanobodies show a diffuse LPL staining. Cells were stained for F-actin (phalloidin 670, far red, shown in grey) and L-plastin (alexa-594, red). LPL Nb5 is shown in green. Pictures were acquired with a confocal laser scanning microscope and are representative for four independent experiments. Bar: 10 µm.

### LPL Nb-expressing THP-1 cells display unstable podosomes with a shorter lifetime

Podosomes are short-lived, with a lifetime of 2–20 minutes [56] and characterized by fast turnover, especially in the leading lamella of cells [57]. Moreover, their inner dynamic is even faster: F-actin in the core turns over 2–3 times during the lifespan of a podosome [2]. We investigated if L-plastin nanobodies affect F-actin turnover and podosome lifetime. Stable THP-1 cells constitutively expressing the F-actin binding peptide LifeAct-mCherry [58] and inducibly expressing EGFP or the EGFP-tagged nanobodies were generated for this purpose. Podosome turnover was investigated by time-lapse imaging of cells for 20 minutes (Fig. 7A and Video S1). THP-1 cells expressing L-plastin Nb5 and 9 did not show a regular cyclic turnover of F-actin in podosomes. The podosomes were very unstable and short-lived, as compared to the other conditions. A significantly larger part of the podosomes of LPL-Nb expressing cells had a lifetime of 0–2 or 2–6 minutes (36–48%), whereas for the other conditions, only 1–14% of the podosomes displayed such short lifespans (Fig. 7B). GSN Nb11-expressing cells on the other hand, display more long-lived podosomes (15–20 minutes) compared to the other conditions, demonstrating a stabilizing effect of this Nb.

**Figure 7:** Podosomes from LPL Nb-expressing cells are dynamically unstable. (A) Stable THP-1 cells constitutively expressing the F-actin binding peptide LifeAct-mCherry and EGFP-tagged LPL Nb5/9, GSN Nb11/13, CapG Nb4 or EGFP were differentiated into macrophages by addition of PMA for 3 days. A 2D reconstruction of podosome turnover in the cells was acquired by time-lapse confocal imaging of life cells for 20 minutes. Actin is shown in red and stable cells in green. The arrow marks the podosome of which the relative actin intensity profile, described in C and D, was determined. Bar: 10 µm. (B) Representation of the average lifetime of podosomes for the different constructs. The lifetime of 120–150 podosomes in 8–12 cells was determined per condition in 3 independent experiments. Error bars represent mean ± SEM. Unpaired t-tests were performed to observe statistical differences between cells expressing EGFP and cells expressing the nanobodies. Statistically significant differences are denoted. (C) Representation of the relative actin intensity profile of a podosome as a function of time for CapG Nb4 (solid line, black), EGFP (dashed line, black), GSN Nb11 (solid line, green), GSN Nb13 (dashed line, green), LPL Nb5 (dashed line, red) and LPL Nb9 (solid line, red). Relative actin intensity profiles were generated for 10–15 podosomes in 5–10 cells per condition. The chosen examples are representative of the generated profiles. (D) Boxplot of the actin intensities (shown in C) for the different constructs. Mann-Whitney Rank Sum tests were performed to observe statistical differences in the distribution of the intensities between cells expressing EGFP and cells expressing nanobodies (ns: non significant p>0.05; * p<0.05; ** p<0.01; *** p<0.001).

The instability of the podosomes of LPL Nb-expressing cells is also apparent when the actin intensity profile is plotted over time (Fig. 7C). Cells expressing EGFP or GSN/CapG nanobodies show a gradual increase and decrease in actin intensity whereas the actin intensities for cells expressing LPL Nb5 and 9 show only slight changes. The podosomes of these cells appear and disappear in such an irregular manner that they cannot be properly formed. Boxplots of the variation in F-actin intensity show significant differences between LPL Nb-expressing cells and cells expressing EGFP or other nanobodies (Fig. 7D). We therefore conclude that plastin nanobodies obstruct formation of new actin bundles leading to podosome instability which results in short-lived podosomes.

## Discussion

The physiological relevance of podosomes in leukocytes has been under considerable investigation in recent years. These intrinsically dynamic structures modulate cellular motility, matrix remodeling and tissue invasion [10]. Impairment of podosome formation leads to a number of symptoms and diseases and the role of actin binding proteins in the maintenance of these structures is also well described (reviewed in [10], [31], [41], [52]). In this study we investigated the effect of nanobodies targeting three well-known actin binding proteins on podosome formation, dynamics and function in macrophage-like THP-1 cells. We observed that CapG is not present in macrophage-differentiated THP-1 podosomes. Expression of CapG Nb4, a high affinity nanobody targeting CapG (Van Impe et al., unpublished data), had no effect whatsoever on podosome formation and function. This nanobody consequently served as a negative control throughout the study.

Whereas CapG does not seem to play any major role in podosome formation, targeting of L-plastin and gelsolin using thoroughly characterized nanobodies demonstrated that L-plastin not only resides in podosomes, but clearly is involved in formation and stability of podosomes. Gelsolin Nb13 is shown here for the first time to trace endogenous gelsolin in a distinct subcellular structure, unlike GSN Nb11. The latter sequesters actin-free gelsolin and perturbs actin binding *in vitro* while GSN Nb13 specifically targets a calcium-activated and actin-bound gelsolin subpopulation but does not inhibit actin binding [40]. This was again confirmed by pull-down experiments in the presence or absence of EGTA performed in this study. Hence, the ability of GSN Nb13 to trace endogenous, actin-bound, gelsolin in podosomes validates our earlier *in vitro* findings asserting that GSN Nb13 does not disturb any apparent function of gelsolin. Moreover, GSN Nb13 is the only nanobody used in this study displaying a podosome-enriched pattern. The *absence* of GSN Nb11 from podosomes further attests that gelsolin is present in an actin-bound configuration in podosomes.

Preventing gelsolin-G-actin interaction (by GSN Nb11) showed no significant effect on podosome formation or function. Earlier studies have demonstrated gelsolin localization in podosomes although its function in that compartment is subject to debate. Gelsolin deficiency in mouse osteoclasts promotes loss of podosomes and actin rings [30]. However, podosome formation in dendritic cells appears to be gelsolin-independent. In osteoclasts, podosomes fuse together into podosome rings or ‘belts’, constituting the sealing zone which is required for bone resorption. Dendritic cells and macrophages generate highly dynamic podosome clusters, changing their location as the cell changes shape whereas the sealing zone is more static [2], [32]. Ma and coworkers suggested that sealing rings may not be derived from podosomes which may explain in part seemingly contradictory data [59]. Functional redundancy is a likely aspect further contributing to the seeming lack of gelsolin involvement in podosome formation or matrix degradation, as observed recently. Indeed, redundancy between gelsolin and supervillin was observed in matrix degradation in human primary macrophages [60]. However, as gelsolin mainly disrupts actin filaments through its F-actin severing activity, its role may differ from plastin and supervillin which both have the ability to bundle actin filaments. Thus, gelsolin could be more involved in renewing the podosome actin pool or actin network destabilization, facilitating actin dynamics, whereas plastin and supervillin can be envisaged as proteins consolidating extant actin filaments. In this respect GSN Nb11 would act as a stabilizer of podosome structure. Life cell imaging indeed demonstrated that the presence of GSN Nb11 in cells, as compared to GSN Nb13 and CapG Nb4, resulted in even more stable and long-lived features although matrix degradation properties remained unmodified.

L-plastin is found in podosomes of human neutrophils [61], adherent macrophages [57], [62] and osteoclasts [63] (reviewed in [42]). L-plastin has been shown to play a regulatory role in formation of the osteoclast sealing ring [59]. At the early phase of bone resorption, actin aggregates are formed which probably serve as precursors for the sealing ring. They speculated that actin aggregates are formed by L-plastin due to its actin bundling capacity. However, L-plastin null osteoclasts demonstrated normal osteoclast differentiation and peripheral podosomes [59].

L-plastin nanobodies were previously shown to perturb immune synapse formation, MTOC docking, proliferation and IL-2 secretion of human T cells, and this was associated with a significant delay in Ser5 L-plastin phosphorylation [38]. Based on the similarities in cytoskeletal architecture between the immune synapse and podosomes [64], we postulated that these nanobodies could affect podosome formation. L-plastin is enriched in podosomes of THP-1 cells and co-localizes with F-actin in these structures. Furthermore, in cells expressing LPL Nb5/9, we were able to discern an increased number of cells lacking podosomes and cells displaying ‘diffuse’ podosomes (blurred phenotype). Importantly, actin turnover in cells expressing these nanobodies was hampered as the podosomes were unstable and short-lived, displaying significantly shorter lifespans compared to the other conditions. A significant decrease the matrix degrading capacity of these cells could be observed.

Podosomes and invadopodia are specialized degrading structures, important for proteolytic cell invasion and matrix remodeling [10], [52]. Podosomes are characterized by a high turnover and are thought to degrade the matrix in a widespread and shallow manner, whereas the more stable invadopodia seem to mediate a more focused and deeper degradation [51]. Production as well as secretion and localization of MMP2, MMP9 and MMP14, were found to be unaffected by nanobody-mediated inhibition of L-plastin. We propose that the defective degrading capacity of these cells is most likely due to structural distortion and malformation of the podosomes, resulting in diminished ECM proteolytic activity. Similar observations have been made in macrophages deficient for the Src family tyrosine kinase Hck. ECM degradation in these cells is impaired, probably as a result of defective podosome rosette formation, since MMP production and secretion are unaffected [65]. Furthermore, MMP activity proves to be subject to regulation itself [52]. For instance, MMP9 activation requires PKCζ [66]. Matrix stiffness also influences proteolytic activity by invadosomes [67]. Several factors therefore seem to be important for proteolytic activity other than mere podosome/invadosome formation.

In leukocytes and macrophages, L-plastin is regulated by Ser5 and Ser7 phosphorylation in the headpiece domain [16], [38], [62], [68]. L-plastin phosphorylation is triggered in response to signals mediating immune response formation, cell migration and proliferation, resulting in relocation of L-plastin to sites of actin assembly [16], [69]. Here we show that phosphorylated L-plastin is enriched in podosomes where it colocalizes with F-actin, consistent with the idea that its phosphorylation enhances F-actin binding and bundling [16], [38].

L-plastin inhibition in THP-1 cells had no effect on LPL phosphorylation, induced by PMA. In a previous study on immune synapse formation between human T cells and antigen presenting cells, we noticed a delay and reduction in LPL phosphorylation upon LPL Nb expression, elicited by CD3/CD28 stimulation [38]. Different phosphorylation stimuli probably trigger diverse signaling pathways leading to LPL phosphorylation. LPL phosphorylation in this study is however not responsible for the observed disruption of podosome stability since no changes in the level or kinetics of L-plastin phosphorylation were noticed.

Direct inhibition of F-actin bundling (LPL Nb5) or preventing L-plastin activation (LPL Nb9) leads to drastic podosome instability over time. Immunoprecipitation experiments in THP-1 cells (this study) or T cells [38] confirm that LPL Nb5 and 9 target an L-plastin population that is actin-free, establishing that these nanobodies act as potent inhibitors. In effect, an earlier study showed complete inhibition of L-plastin activity at equimolar ratios with the respective nanobodies [39]. These molecules very likely perturb the equilibrium between inactive and active L-plastin, making the latter unavailable for F-actin binding and bundling, leading to defected podosome (core) formation in THP-1 cells. Podosomes in macrophages are especially dynamic and they undergo 2 overlaying cycles of stiffness, which may correspond to actin filament turnover and bundling [70].

Apart from L-plastin, other actin bundling and cross-linking proteins participate in podosome formation and/or matrix degradation, including alpha-actinin [71], filamin A [72], fascin [73] and supervillin [60]. Actin bundling by fascin is required for invadopodia formation [74]. Li and coworkers further demonstrated that although fascin does affect the lifespan of invadopodia, it seems not to be required for bundling of rapidly cycling actin since the turnover rate of actin was unaffacted [74]. This points to a possible role for L-plastin in the bundling of rapidly cycling actin in invadopodia.

The approach used in this study was aimed at blocking discrete biological functions of an endogenous ‘undruggable’ target without manipulating its expression. We have demonstrated that LPL nanobodies represent a valid and powerful tool to unsettle LPL functionality *in vivo* and to highlight its role as a cementing molecule in stabilizing podosomes in macrophage-like THP-1 cells, perturbation of which induced defects in matrix degradation. This study and earlier reports illustrate how nanobodies can be applied in different cellular contexts to investigate various functions of proteins in particular cellular processes. In cytoskeleton studies they have proven helpful in investigating cancer cell invasion and motility [39], [40] (Van Impe et al, unpublished data) as well as studying immunological processes [38]. Nanobodies can be either used as ‘tracers’ with no impact on antigen functionality and/or localization, or as direct protein inhibitors. As such they represent an instrument of choice to mimic the activity of small pharmacological compounds. Such molecules are difficult, albeit not impossible [75]–[77] to raise against structural (non-enzymatic) proteins, many of which play a role in the etiology or progression of various diseases [78].

## Materials and Methods

### Ethics

An ethics statement is not required for this work.

### Reagents and antibodies

A monoclonal anti-V5 antibody was purchased from Invitrogen (Merelbeke, Belgium); monoclonal L-plastin antibody was from Thermo Scientific Lab Vison (Kalamazoo, MI, USA). Gelsolin monoclonal antibody and DAPI were from Sigma-Aldrich (St. Louis, MO, USA). Polyclonal anti-gelsolin, anti-CapG and anti-EGFP antibodies were obtained as described [26], [79]. Polyclonal rabbit IgG against serine-5 phosphorylated L-plastin (anti-Ser5-P) was a kind gift from dr. Evelyne Friedrich (University of Luxembourg) and has been characterized before [16]. Rabbit anti-EGFP antibody was purchased from Cell Signaling (Danvers, MA, USA). Alexa Fluor 488/594-conjugated goat anti-mouse/anti-rabbit IgGs and Alexa Fluor 594 phalloidin were obtained from Molecular Probes®-Life Technologies™ (Grand Island, NY, USA). Acti-stain™ 670 phalloidin was from Tebu-Bio (Le Perray-en-Yvelines, France). Rabbit monoclonal anti-MMP2, MMP9 and MMP14 (MT1-MMP) were purchased from Epitomics (Burlingame, CA, USA). Rabbit polyclonal MMP2 was from Santa Cruz Biotechnology (Dallas, Texas, USA). A cortactin monoclonal antibody and the QCM™ Gelatin Invadopodia Assay containing Cy3-labeled gelatin, were purchased from Millipore (Billerica, MA, USA). Phorbol 12-myristate 13-acetate (PMA), fibronectin and gelatin were from Sigma-Aldrich (St. Louis, MO, USA). Doxycycline was from Clontech (Mountain View, CA, USA). Amaxa® Cell Line Nucleofector® Kit V was obtained from Lonza (Cologne, Germany).

### Cell culture and transfection

THP-1 monocytic leukemia cells (ATCC® TIB-202™) were maintained at 37°C in a humidified 5% CO_2_ incubator and grown in RPMI 1640 (Gibco®- Life Technologies™, Grand Island, NY, USA) supplemented with 10% fetal bovine serum, 0.1% (0.05 mM) beta-mercaptoethanol, 100 µg/ml streptomycin and 100 IU/ml penicillin. THP-1 cells were differentiated into adherent, macrophage-like THP-1 cells by stimulation with 350 nM PMA for 3 days.

### Generation of nanobodies and cDNA cloning

L-plastin and gelsolin nanobodies were obtained in collaboration with the VIB nanobody service facility and described earlier [39], [40]. The Actin-mCherry was kindly provided by dr. Klemens Rottner (Helmholtz Centre for Infection Research, Braunschweig, Germany).

### Generation of stable THP-1 cell lines

THP-1 cells stably expressing EGFP or EGFP-tagged (LPL/GSN/CapG) nanobodies were created using the Lenti-X™ Tet-On^R^ Advanced Inducible Expression System from Clontech (Mountain View, CA, USA). Upon transduction, 12-well plates were coated with fibronectin, after which 500,000 cells and viral mixture (MOI: 20) in a total amount of 1 ml were added. Cells were then centrifuged for one hour at 1500 rpm. Nanobodies and EGFP were cloned in the pLVX-Tight-Puro vector. Expression of nanobodies/EGFP was induced by stimulation with 500 ng/ml doxycycline for 24–48 h. For live cell imaging, these cells were additionally transduced with the F-actin probe Lifeact-mCherry [58], which was constitutively expressed. Lifeact-mCherry virus was a kind gift from dr. Isabelle Maridonneau-Parini (Institut de Pharmacologie et de Biologie Structurale, University of Toulouse, France).

### Immunoprecipitation and immunoblotting

Immunoprecipitation and immunoblotting experiments were performed as described before [38].

### Immunostaining and microscopy

Immunostaining experiments were performed as described before [38]. Stained cells were analyzed using a Carl Zeiss Axiovert 200 M Apotome epifluorescence microscope or an Olympus IX-81 laser scanning confocal microscope. The Zeiss epifluorescence microsope is equipped with an Axiocam cooled charge-coupled device (CCD) camera and data processing was done with Axiovision software (Zeiss). The Olympus confocal microscope is equipped with a motorized stage and an incubator chamber to maintain the temperature and CO_2_ concentration constant. Analysis of images, including generation of intensity profiles, was done with Fluoview 1000 software.

### Matrix degradation assay

Coverslips were coated with Cy3-labeled gelatin according to the manufacturer's instructions. 160,000 PMA-differentiated macrophage-like THP-1-Nb cells were seeded onto the gelatin-coated coverslips for 24 h at 37°C. The cells were subsequently fixed and nuclei were stained with DAPI (0.4 µg/ml). Dark holes in the matrix correspond to degraded gelatin; these cells were counted as ‘degrading cells’.

### Zymography

300,000–400,000 PMA-differentiated macrophage-like THP-1-Nb cells were plated in uncoated or fibronectin-coated 12-well plates. After 24 h, growth medium was substituted for serum-free medium, supplemented with PMA and doxycycline. Another 24 h later, medium was collected and boiled with non-reducing SDS-PAGE buffer. Sample proteins were separated on 10% acrylamide/0.075% gelatin gels, after which the gels were soaked in 2% Triton X-100 for 1 h to remove the SDS and to allow protein renaturation. The gels were rinsed once with MQ and incubated in substrate buffer (0.05 M Tris-HCl, pH 7.5, 5 mM CaCl_2_, 0.02% (w/v) NaN_3_) at 37°C overnight. After incubation the gels were stained with Coomassie Brilliant Blue R-250 for 20 minutes, followed by incubation in destaining solution (20% methanol/10% acetic acid) until proteolytic activity could be resolved.

### Phosphorylation assay

THP-1-Nb cells were stimulated with 350 nM PMA for the times indicated. Following stimulation, cells were lysed and subjected to SDS-PAGE and western blotting.

### Live cell imaging of podosome turnover

440,000 THP-1 cells, constitutively expressing LifeAct-mCherry, were seeded in 35 mm μ-dishes from Ibidi (Planegg/Martinsried, Germany). After stimulation with PMA and doxycycline, the macrophage-like THP-1-Nb-LifeAct cells were imaged using the Olympus confocal microscope, at a constant temperature of 37°C. In each experiment, time-lapse images of the live cells were acquired every 20 seconds in one z plane over a period of 20 minutes, resulting in a 2D reconstruction of the actin turnover in the podosomes. Subsequently, relative actin intensity profiles as a function of time were generated for representative podosomes of each condition. A line was drawn across the podosome, followed by analysis of the intensity of the actin staining along that line (Fluoview 1000 software: ‘line series analysis’). These intensities were then plotted as a function of time.

### Statistical analysis

Statistical analysis was performed with Unpaired Student *t* tests or Mann-Whitney Rank Sum tests, when samples were normally or not normally distributed respectively (SigmaPlot 12).

## Supporting Information

Figure S1 **GSN Nb13 is enriched in podosomes of PMA-stimulated THP-1 cells.** Representation of the relative GFP, LPL or GSN and actin intensity profiles of the cells, shown in Fig. 3 of the manuscript. The intensity profiles are presented as function of the length, measured along a line, intersecting the (podosomes of the) cell.
(TIF)

Figure S2 **Expression of LPL/GSN/CapG nanobodies does not alter the production, secretion or localization of MMPs.** (A) Stably transduced THP-1 cells (5×10^5^ cells per condition) were seeded into fibronectin-coated 12-wells in the presence of PMA for 72 h. Conditioned media of these cells were collected and subjected to gelatin zymography. (B) Immunoblot analysis was performed on these media for (pro-)MMP2. These data are representative of 2–3 independent experiments. (C, D) Parental (C) and stably transduced (D) THP-1 cells were plated onto coverslips and differentiated to macrophages by PMA. These cells were then stained for MMP2, MMP9 or MMP14 (alexa 594, red); L-plastin (alexa 488, green) and F-actin (phalloidin 670, far red, shown in grey). Cells expressing EGFP-tagged nbs are shown in green (D). The pictures were acquired with a laser scanning confocal microscope and are representative for two independent experiments. Bar: 10 µm.
(TIF)

Figure S3 **LPL Nbs disturb podosome integrity.** Confocal images showing the different phenotypes, observed in THP-1 macrophages. Cells expressing CapG Nb4 or LPL Nb5 are shown in green and cells were stained for cortactin (alexa 594, red) and F-actin (phalloidin 670, far red, shown in grey). Pictures were acquired with a confocal laser scanning microscope and are representative for two independent experiments. Bar: 10 µm.
(TIF)

Video S1 **LPL Nb-expressing macrophages are unable to form stable podosomes.** Stable THP-1 cells constitutively expressing LifeAct-Cherry and inducibly expressing EGFP (A) or EGFP-tagged CapG Nb4 (B), GSN Nb11/13 (C/D) or LPL Nb5/9 (E/F), were differentiated into macrophages by adding PMA for 3 days. A 2D reconstruction of podosome turnover in cells was acquired by time-lapse confocal imaging of live cells for 20 minutes. Actin is shown in red and EGFP or the respective nanobodies in green. LPL-Nb THP-1 cells are characterized by a higher podosome turnover compared to other nanobodies, or the EGFP control. Bar: 10 µm.
(ZIP)

## References

[1] BurnsS, ThrasherAJ, BlundellMP, MacheskyL, JonesGE (2001) Configuration of human dendritic cell cytoskeleton by Rho GTPases, the WAS protein, and differentiation. Blood 98: 1142–1149.1149346310.1182/blood.v98.4.1142

[2] DestaingO, SaltelF, GeminardJC, JurdicP, BardF (2003) Podosomes display actin turnover and dynamic self-organization in osteoclasts expressing actin-green fluorescent protein. Mol Biol Cell 14: 407–416.1258904310.1091/mbc.E02-07-0389PMC149981

[3] LinderS, NelsonD, WeissM, AepfelbacherM (1999) Wiskott-Aldrich syndrome protein regulates podosomes in primary human macrophages. Proc Natl Acad Sci U S A 96: 9648–9653.1044974810.1073/pnas.96.17.9648PMC22264

[4] OsiakAE, ZennerG, LinderS (2005) Subconfluent endothelial cells form podosomes downstream of cytokine and RhoGTPase signaling. Exp Cell Res 307: 342–353.1589431310.1016/j.yexcr.2005.03.035

[5] VaronC, TatinF, MoreauV, Van Obberghen-SchillingE, Fernandez-SauzeS, et al (2006) Transforming growth factor beta induces rosettes of podosomes in primary aortic endothelial cells. Mol Cell Biol 26: 3582–3594.1661199810.1128/MCB.26.9.3582-3594.2006PMC1447430

[6] HaiCM, HahneP, HarringtonEO, GimonaM (2002) Conventional protein kinase C mediates phorbol-dibutyrate-induced cytoskeletal remodeling in a7r5 smooth muscle cells. Exp Cell Res 280: 64–74.1237234010.1006/excr.2002.5592

[7] TatinF, VaronC, GenotE, MoreauV (2006) A signalling cascade involving PKC, Src and Cdc42 regulates podosome assembly in cultured endothelial cells in response to phorbol ester. J Cell Sci 119: 769–781.1644932110.1242/jcs.02787

[8] WeaverAM (2006) Invadopodia: specialized cell structures for cancer invasion. Clin Exp Metastasis 23: 97–105.1683022210.1007/s10585-006-9014-1

[9] CalleY, BurnsS, ThrasherAJ, JonesGE (2006) The leukocyte podosome. Eur J Cell Biol 85: 151–157.1654655710.1016/j.ejcb.2005.09.003

[10] LinderS, AepfelbacherM (2003) Podosomes: adhesion hot-spots of invasive cells. Trends Cell Biol 13: 376–385.1283760810.1016/s0962-8924(03)00128-4

[11] OchsHD (2001) The Wiskott-Aldrich syndrome. Clin Rev Allergy Immunol 20: 61–86.1126922910.1385/CRIAI:20:1:61

[12] LuxenburgC, GeblingerD, KleinE, AndersonK, HaneinD, et al (2007) The architecture of the adhesive apparatus of cultured osteoclasts: from podosome formation to sealing zone assembly. PLoS One 2: e179.1726488210.1371/journal.pone.0000179PMC1779809

[13] LeavittJ (1994) Discovery and characterization of two novel human cancer-related proteins using two-dimensional gel electrophoresis. Electrophoresis 15: 345–357.805586510.1002/elps.1150150154

[14] ParkT, ChenZP, LeavittJ (1994) Activation of the leukocyte plastin gene occurs in most human cancer cells. Cancer Res 54: 1775–1781.8137292

[15] NambaY, ItoM, ZuY, ShigesadaK, MaruyamaK (1992) Human T cell L-plastin bundles actin filaments in a calcium-dependent manner. J Biochem 112: 503–507.149100510.1093/oxfordjournals.jbchem.a123929

[16] JanjiB, GigantiA, De CorteV, CatillonM, BruyneelE, et al (2006) Phosphorylation on Ser5 increases the F-actin-binding activity of L-plastin and promotes its targeting to sites of actin assembly in cells. J Cell Sci 119: 1947–1960.1663607910.1242/jcs.02874

[17] KhuranaS, GeorgeSP (2008) Regulation of cell structure and function by actin-binding proteins: villin's perspective. FEBS Lett 582: 2128–2139.1830799610.1016/j.febslet.2008.02.040PMC2680319

[18] YinHL, StosselTP (1979) Control of cytoplasmic actin gel-sol transformation by gelsolin, a calcium-dependent regulatory protein. Nature 281: 583–586.49232010.1038/281583a0

[19] YinHL, StosselTP (1980) Purification and structural properties of gelsolin, a Ca2+-activated regulatory protein of macrophages. J Biol Chem 255: 9490–9493.6251090

[20] YoungCL, SouthwickFS, WeberA (1990) Kinetics of the interaction of a 41-kilodalton macrophage capping protein with actin: promotion of nucleation during prolongation of the lag period. Biochemistry 29: 2232–2240.233760110.1021/bi00461a005

[21] YuFX, JohnstonPA, SudhofTC, YinHL (1990) gCap39, a calcium ion- and polyphosphoinositide-regulated actin capping protein. Science 250: 1413–1415.225591210.1126/science.2255912

[22] SilacciP, MazzolaiL, GauciC, StergiopulosN, YinHL, et al (2004) Gelsolin superfamily proteins: key regulators of cellular functions. Cell Mol Life Sci 61: 2614–2623.1552616610.1007/s00018-004-4225-6PMC11924436

[23] CooperJA, SchaferDA (2000) Control of actin assembly and disassembly at filament ends. Curr Opin Cell Biol 12: 97–103.1067935810.1016/s0955-0674(99)00062-9

[24] WitkeW, LiW, KwiatkowskiDJ, SouthwickFS (2001) Comparisons of CapG and gelsolin-null macrophages: demonstration of a unique role for CapG in receptor-mediated ruffling, phagocytosis, and vesicle rocketing. J Cell Biol 154: 775–784.1151459110.1083/jcb.200101113PMC2196452

[25] De CorteV, BruyneelE, BoucherieC, MareelM, VandekerckhoveJ, et al (2002) Gelsolin-induced epithelial cell invasion is dependent on Ras-Rac signaling. EMBO J 21: 6781–6790.1248599910.1093/emboj/cdf680PMC139100

[26] Van den AbbeeleA, De CorteV, Van ImpeK, BruyneelE, BoucherieC, et al (2007) Downregulation of gelsolin family proteins counteracts cancer cell invasion in vitro. Cancer Lett 255: 57–70.1749374610.1016/j.canlet.2007.03.023

[27] ParikhSS, LitherlandSA, Clare-SalzlerMJ, LiW, GuligPA, et al (2003) CapG(−/−) mice have specific host defense defects that render them more susceptible than CapG(+/+) mice to Listeria monocytogenes infection but not to Salmonella enterica serovar Typhimurium infection. Infect Immun 71: 6582–6590.1457368010.1128/IAI.71.11.6582-6590.2003PMC219612

[28] SunHQ, KwiatkowskaK, WootenDC, YinHL (1995) Effects of CapG overexpression on agonist-induced motility and second messenger generation. J Cell Biol 129: 147–156.769898110.1083/jcb.129.1.147PMC2120377

[29] ChellaiahM, FitzgeraldC, AlvarezU, HruskaK (1998) c-Src is required for stimulation of gelsolin-associated phosphatidylinositol 3-kinase. J Biol Chem 273: 11908–11916.956561810.1074/jbc.273.19.11908

[30] ChellaiahM, KizerN, SilvaM, AlvarezU, KwiatkowskiD, et al (2000) Gelsolin deficiency blocks podosome assembly and produces increased bone mass and strength. J Cell Biol 148: 665–678.1068424910.1083/jcb.148.4.665PMC2169374

[31] LinderS, KoppP (2005) Podosomes at a glance. J Cell Sci 118: 2079–2082.1589098210.1242/jcs.02390

[32] HammarfjordO, FaletH, GurniakC, HartwigJH, WallinRP (2011) Gelsolin-independent podosome formation in dendritic cells. PLoS One 6: e21615.2177933010.1371/journal.pone.0021615PMC3136926

[33] HarmsenMM, De HaardHJ (2007) Properties, production, and applications of camelid single-domain antibody fragments. Appl Microbiol Biotechnol 77: 13–22.1770491510.1007/s00253-007-1142-2PMC2039825

[34] Van BockstaeleF, HolzJB, RevetsH (2009) The development of nanobodies for therapeutic applications. Curr Opin Investig Drugs 10: 1212–1224.19876789

[35] HmilaI, SaerensD, Ben AbderrazekR, VinckeC, AbidiN, et al (2010) A bispecific nanobody to provide full protection against lethal scorpion envenoming. FASEB J 24: 3479–3489.2041044310.1096/fj.09-148213

[36] RasmussenSG, DeVreeBT, ZouY, KruseAC, ChungKY, et al (2011) Crystal structure of the beta2 adrenergic receptor-Gs protein complex. Nature 477: 549–555.2177228810.1038/nature10361PMC3184188

[37] HultbergA, TempertonNJ, RosseelsV, KoendersM, Gonzalez-PajueloM, et al (2011) Llama-derived single domain antibodies to build multivalent, superpotent and broadened neutralizing anti-viral molecules. PLoS One 6: e17665.2148377710.1371/journal.pone.0017665PMC3069976

[38] De ClercqS, ZwaenepoelO, MartensE, VandekerckhoveJ, GuillabertA, et al (2013) Nanobody-induced perturbation of LFA-1/L-plastin phosphorylation impairs MTOC docking, immune synapse formation and T cell activation. Cell Mol Life Sci 70: 909–922.2300101210.1007/s00018-012-1169-0PMC11113607

[39] DelanoteV, VanlooB, CatillonM, FriederichE, VandekerckhoveJ, et al (2010) An alpaca single-domain antibody blocks filopodia formation by obstructing L-plastin-mediated F-actin bundling. FASEB J 24: 105–118.1972675610.1096/fj.09-134304

[40] Van den AbbeeleA, De ClercqS, De GanckA, De CorteV, Van LooB, et al (2010) A llama-derived gelsolin single-domain antibody blocks gelsolin-G-actin interaction. Cell Mol Life Sci 67: 1519–1535.2014075010.1007/s00018-010-0266-1PMC11115616

[41] BuccioneR, OrthJD, McNivenMA (2004) Foot and mouth: podosomes, invadopodia and circular dorsal ruffles. Nat Rev Mol Cell Biol 5: 647–657.1536670810.1038/nrm1436

[42] MorleySC (2012) The actin-bundling protein L-plastin: a critical regulator of immune cell function. Int J Cell Biol 2012: 935173.2219475010.1155/2012/935173PMC3238366

[43] AuwerxJ (1991) The human leukemia cell line, THP-1: a multifacetted model for the study of monocyte-macrophage differentiation. Experientia 47: 22–31.199923910.1007/BF02041244

[44] TsuchiyaS, YamabeM, YamaguchiY, KobayashiY, KonnoT, et al (1980) Establishment and characterization of a human acute monocytic leukemia cell line (THP-1). Int J Cancer 26: 171–176.697072710.1002/ijc.2910260208

[45] AbrinkM, GoblAE, HuangR, NilssonK, HellmanL (1994) Human cell lines U-937, THP-1 and Mono Mac 6 represent relatively immature cells of the monocyte-macrophage cell lineage. Leukemia 8: 1579–1584.8090034

[46] TsuchiyaS, KobayashiY, GotoY, OkumuraH, NakaeS, et al (1982) Induction of maturation in cultured human monocytic leukemia cells by a phorbol diester. Cancer Res 42: 1530–1536.6949641

[47] TsuboiS (2007) Requirement for a complex of Wiskott-Aldrich syndrome protein (WASP) with WASP interacting protein in podosome formation in macrophages. J Immunol 178: 2987–2995.1731214410.4049/jimmunol.178.5.2987PMC1855218

[48] BurgerKL, DavisAL, IsomS, MishraN, SealsDF (2011) The podosome marker protein Tks5 regulates macrophage invasive behavior. Cytoskeleton (Hoboken) 68: 694–711.2202121410.1002/cm.20545PMC3240724

[49] KellyT, MuellerSC, YehY, ChenWT (1994) Invadopodia promote proteolysis of a wide variety of extracellular matrix proteins. J Cell Physiol 158: 299–308.810656710.1002/jcp.1041580212

[50] YamaguchiH, PixleyF, CondeelisJ (2006) Invadopodia and podosomes in tumor invasion. Eur J Cell Biol 85: 213–218.1654656310.1016/j.ejcb.2005.10.004

[51] LinderS (2007) The matrix corroded: podosomes and invadopodia in extracellular matrix degradation. Trends Cell Biol 17: 107–117.1727530310.1016/j.tcb.2007.01.002

[52] LinderS, WiesnerC, HimmelM (2011) Degrading devices: invadosomes in proteolytic cell invasion. Annu Rev Cell Dev Biol 27: 185–211.2180101410.1146/annurev-cellbio-092910-154216

[53] DreierR, GrässelS, FuchsS, SchaumburgerJ, BrucknerP (2004) Pro-MMP-9 is a specific macrophage product and is activated by osteoarthritic chondrocytes via MMP-3 or a MT1-MMP/MMP-13 cascade. Exp Cell Res 297: 303–312.1521293610.1016/j.yexcr.2004.02.027

[54] Banon-RodriguezI, MonypennyJ, RagazziniC, FrancoA, CalleY, et al (2011) The cortactin-binding domain of WIP is essential for podosome formation and extracellular matrix degradation by murine dendritic cells. Eur J Cell Biol 90: 213–223.2095209310.1016/j.ejcb.2010.09.001

[55] EsparzaJ, VilardellC, CalvoJ, JuanM, VivesJ, et al (1999) Fibronectin upregulates gelatinase B (MMP-9) and induces coordinated expression of gelatinase A (MMP-2) and its activator MT1-MMP (MMP-14) by human T lymphocyte cell lines. A process repressed through RAS/MAP kinase signaling pathways. Blood 94: 2754–2766.10515879

[56] MurphyDA, CourtneidgeSA (2011) The ‘ins’ and ‘outs’ of podosomes and invadopodia: characteristics, formation and function. Nat Rev Mol Cell Biol 12: 413–426.2169790010.1038/nrm3141PMC3423958

[57] EvansJG, CorreiaI, KrasavinaO, WatsonN, MatsudairaP (2003) Macrophage podosomes assemble at the leading lamella by growth and fragmentation. J Cell Biol 161: 697–705.1275623710.1083/jcb.200212037PMC2199349

[58] RiedlJ, CrevennaAH, KessenbrockK, YuJH, NeukirchenD, et al (2008) Lifeact: a versatile marker to visualize F-actin. Nat Methods 5: 605–607.1853672210.1038/nmeth.1220PMC2814344

[59] MaT, SadashivaiahK, MadayiputhiyaN, ChellaiahMA (2010) Regulation of sealing ring formation by L-plastin and cortactin in osteoclasts. J Biol Chem 285: 29911–29924.2065088810.1074/jbc.M109.099697PMC2943304

[60] BhuwaniaR, CornfineS, FangZ, KrugerM, LunaEJ, et al (2012) Supervillin couples myosin-dependent contractility to podosomes and enables their turnover. J Cell Sci 125: 2300–2314.2234426010.1242/jcs.100032PMC3367944

[61] JonesSL, BrownEJ (1996) FcgammaRII-mediated adhesion and phagocytosis induce L-plastin phosphorylation in human neutrophils. J Biol Chem 271: 14623–14630.866306610.1074/jbc.271.24.14623

[62] MessierJM, ShawLM, ChafelM, MatsudairaP, MercurioAM (1993) Fimbrin localized to an insoluble cytoskeletal fraction is constitutively phosphorylated on its headpiece domain in adherent macrophages. Cell Motil Cytoskeleton 25: 223–233.822190010.1002/cm.970250303

[63] BabbSG, MatsudairaP, SatoM, CorreiaI, LimSS (1997) Fimbrin in podosomes of monocyte-derived osteoclasts. Cell Motil Cytoskeleton 37: 308–325.925850410.1002/(SICI)1097-0169(1997)37:4<308::AID-CM3>3.0.CO;2-0

[64] WernimontSA, CortesioCL, SimonsonWT, HuttenlocherA (2008) Adhesions ring: a structural comparison between podosomes and the immune synapse. Eur J Cell Biol 87: 507–515.1834353010.1016/j.ejcb.2008.01.011PMC2570187

[65] CougouleC, Le CabecV, PoinclouxR, Al SaatiT, MegeJL, et al (2010) Three-dimensional migration of macrophages requires Hck for podosome organization and extracellular matrix proteolysis. Blood 115: 1444–1452.1989757610.1182/blood-2009-04-218735PMC5070714

[66] XiaoH, BaiXH, KapusA, LuWY, MakAS, et al (2010) The protein kinase C cascade regulates recruitment of matrix metalloprotease 9 to podosomes and its release and activation. Mol Cell Biol 30: 5545–5561.2093777510.1128/MCB.00382-10PMC2976425

[67] AlexanderNR, BranchKM, ParekhA, ClarkES, IwuekeIC, et al (2008) Extracellular matrix rigidity promotes invadopodia activity. Curr Biol 18: 1295–1299.1871875910.1016/j.cub.2008.07.090PMC2555969

[68] ShinomiyaH, HagiA, FukuzumiM, MizobuchiM, HirataH, et al (1995) Complete primary structure and phosphorylation site of the 65-kDa macrophage protein phosphorylated by stimulation with bacterial lipopolysaccharide. J Immunol 154: 3471–3478.7897227

[69] Al TanouryZ, Schaffner-ReckingerE, HalavatyiA, HoffmannC, MoesM, et al (2010) Quantitative kinetic study of the actin-bundling protein L-plastin and of its impact on actin turn-over. PLoS One 5: e9210.2016915510.1371/journal.pone.0009210PMC2821400

[70] LabernadieA, ThibaultC, VieuC, Maridonneau-PariniI, CharriereGM (2010) Dynamics of podosome stiffness revealed by atomic force microscopy. Proc Natl Acad Sci U S A 107: 21016–21021.2108169910.1073/pnas.1007835107PMC3000246

[71] LuxenburgC, Winograd-KatzS, AddadiL, GeigerB (2012) Involvement of actin polymerization in podosome dynamics. J Cell Sci 125: 1666–1672.2232850710.1242/jcs.075903PMC3346827

[72] GuietR, VerolletC, LamsoulI, CougouleC, PoinclouxR, et al (2012) Macrophage mesenchymal migration requires podosome stabilization by filamin A. J Biol Chem 287: 13051–13062.2233468810.1074/jbc.M111.307124PMC3339984

[73] YamakitaY, MatsumuraF, LipscombMW, ChouPC, WerlenG, et al (2011) Fascin1 promotes cell migration of mature dendritic cells. J Immunol 186: 2850–2859.2126306810.4049/jimmunol.1001667PMC3526951

[74] LiA, DawsonJC, Forero-VargasM, SpenceHJ, YuX, et al (2010) The actin-bundling protein fascin stabilizes actin in invadopodia and potentiates protrusive invasion. Curr Biol 20: 339–345.2013795210.1016/j.cub.2009.12.035PMC3163294

[75] RizviSA, NeidtEM, CuiJ, FeigerZ, SkauCT, et al (2009) Identification and characterization of a small molecule inhibitor of formin-mediated actin assembly. Chem Biol 16: 1158–1168.1994213910.1016/j.chembiol.2009.10.006PMC2784894

[76] GauvinTJ, FukuiJ, PetersonJR, HiggsHN (2009) Isoform-selective chemical inhibition of mDia-mediated actin assembly. Biochemistry 48: 9327–9329.1976470810.1021/bi901354zPMC2758331

[77] NolenBJ, TomasevicN, RussellA, PierceDW, JiaZ, et al (2009) Characterization of two classes of small molecule inhibitors of Arp2/3 complex. Nature 460: 1031–1034.1964890710.1038/nature08231PMC2780427

[78] Van AudenhoveI, Van ImpeK, Ruano-GallegoD, De ClercqS, De MuynckK, et al (2013) Mapping cytoskeletal protein function in cells by means of nanobodies. Cytoskeleton doi:10.1002/cm.21122 10.1002/cm.2112223818458

[79] IrobiJ, Van ImpeK, SeemanP, JordanovaA, DierickI, et al (2004) Hot-spot residue in small heat-shock protein 22 causes distal motor neuropathy. Nat Genet 36: 597–601.1512225310.1038/ng1328

